# Intraoperative Cryoprecipitate Transfusion and Its Association with the Incidence of Biliary Complications after Liver Transplantation-A Retrospective Cohort Study

**DOI:** 10.1371/journal.pone.0060727

**Published:** 2013-05-10

**Authors:** Shuang Liu, Junwei Fan, Xiaoliang Wang, Zijun Gong, Shuyun Wang, Li Huang, Tonghai Xing, Tao Li, Zhihai Peng, Xing Sun

**Affiliations:** Department of General Surgery, Shanghai First People's Hospital, School of Medicine, Shanghai Jiao Tong University, Shanghai, China; Cardiff University, United Kingdom

## Abstract

**Background:**

Cryoprecipitate is largely used for acquired hypofibrinogenemia in the setting of massive hemorrhage in liver transplantation (LT). However, the influence of intraoperative cryoprecipitate transfusion on biliary complications (BC) after LT has not been studied in detail.

**Study Design and Methods:**

In a series of 356 adult patients who received their first LT, the causes of BC were retrospectively studied by multivariate logistic regression analysis. The clinical relationship between intraoperative cryoprecipitate transfusion and BC occurrence was studied through a retrospective cohort study in patients. All patients received follow-ups for one year, and, during the follow-up period, the time of BC occurrence and liver biopsies were recorded.

**Results:**

Intraoperative cryoprecipitate transfusion (RR = 3.46, 95% CI [1.72–6.97], P<0.001), cold ischemia time >8 h (RR = 4.24, 95% CI [2.28–7.92], P<0.01), and high-level Child-Pugh ( RR = 1.71, 95% CI [1.11–2.63], P = 0.014) are independent risk factors to predict BC after LT according to time-to-event analysis. One year BC-free survival probability of patients received intraoperative cryoprecipitate transfusions was significantly lower when compared to the group that received no cryoprecipitate(P<0.001). Moreover, BC patients in the cryoprecipitate transfusion group owned different liver pathological feature, pathological micro-thrombus formation and cholestasis were seen more often (41.4% vs 0%, 62.1% vs 12.5%, respectively) than no cryoprecipitate transfusion group.

**Conclusion:**

These findings suggested that intraoperative cryoprecipitate transfusion was associated with BC after LT. The mechanism of BC occurrence might involve micro-thrombus formation and immune rejection.

## Introduction

Improvement of surgical techniques and immunosuppression, as well as better organ preservation have brought great improvements in success rate of liver transplantation (LT). However, postoperative biliary complications (BC) remain the weakest part of LT, and have been referred to as the “Achilles' heel” of the procedure [1]. According to the literature, the incidence of BC after LT varies from 10% to 30% [2], [3].

Although BC is a significant source of patient morbidity and mortality after LT, the mechanism of BC remains unclear and identifying risk factors of BC might give insight into the pathogenesis and reduce graft loss. Due to improvement in surgical techniques and perioperative care, the incidence of biliary anastomosis strictures and leaks decreased, however the incidence of non-anastomotic bile duct stricture became more apparent [4], [5]. Previous studies in LT have found that apart from the obvious life-saving benefits, an increase in blood loss and subsequent transfusion of blood products has been associated with substantial side effects, such as increased risk of BC [6] [7].

Cryoprecipitate provided a major therapeutic advantage for patients in LT, as it does not require blood cross- matching, and is convenient to obtain. Currently, the most common indication for the use of this product is in hypofibrinogenemia in the setting of massive hemorrhage. With its increased usage in surgery, there has also been a high incidence of inappropriate use of cryoprecipitate which may range from 24%–62% [8], [9]. The influence of intraoperative cryoprecipitate transfusion on BC after LT, however, has not been studied in detail.

We retrospectively reviewed our LT patients in a single center to address two issues. Firstly, whether or not intraoperative cryoprecipitate transfusion is associated with BC after LT. If this was the case, our second objective was to detect the possible mechanism of BC occurrence. This information would allow the implementation of specific measures in high-risk patients to minimize BC occurrence.

## Materials and Methods

### Patients

389 patients who underwent LT at Shanghai First People's Hospital between January 1, 2005 and December 31, 2010 were initially selected. All transplants were from cardiac death donors. We excluded Data from children (n = 1), patients who required re-transplantation (n = 23), paients with primary biliary cirrhosis (n = 7) and primary sclerosing cholangitis (n = 2), and the remaining 356 consecutive adult cases formed the analysis population.

We defined BC on the basis of a 2-fold increase of serum bilirubin greater than normal levels occurring within the first year after LT. The increased serum bilirubin levels also needed to be sustained for at least 1 week. The final diagnosis of BC was then verified through “gold standard” protocols as follows : magnetic resonance cholangiopancreatography (MRCP), endoscopic retrograde cholangio-pancreatography(ERCP), percutaneous transhepatic cholangiography(PTC), liver biopsy or intraoperative observation. The biliary anastomotic strictures and vascular anastomotic stenosis were not included in this study.

In our center, we apply cryoprecipitate transfusion to patients with fibrinogen <1.0 g/l or patients with significant coagulation problems (prothrombin time >6 s), to compensate fibrinogen or coagulation factors. We'll stop transfusion when the thrombelastography during surgery recovers to normal range or blood exudation is significantly improved. For patients with large amount of blood loss (>2500 ml), we'll have to transfuse blood cells which will very often lead to decreased fibrinogen (<1 g/l) and lead to cryo transfusion. For some patients with coagulation problems, even when the blood loss is less than 2500 ml, we need to do cryo transfusion to improve their coagulation function to facilitate the operation.

Clinical characteristics of these patients, including donor and recipient variables, as well as surgical factors were obtained from the China Liver Transplantation Registry (CTLR) computer database. When necessary, the original patient notes were reviewed for missing information. Risk factors determined to be meaningful predictors of BC were selected based on a review of the literature. National legislation and the ethical committee of Shanghai First People's Hospital approved this retrospective study.

### Surgical techniques and perioperative care

Grafts from cardiac death donors were used for all patients. The orthotropic LT technique was used for implantation. In our center, duct-to-duct reconstruction for biliary anastomosis using 7/0 prolene sutures was performed with microsurgical technique without a stent or T-tube. All surgical procedures were supervised by one of the two most experienced surgeons, who assume responsibility for the surgical team. Color Doppler sonographer was used for detecting abnormalities of the hepatic vasculature in patients with LT in the first 3 days. All patients were treated with standard immunosuppressive therapy as described elsewhere [10]. Anesthetic management during LT was performed using a common protocol previously decided by consensus. During the research period, the anesthetic protocol had little substantive change.

### Follow up

Follow-ups were performed every week in the first three months, then fortnightly until six months post-transplant. Beyond this, follow-ups were performed monthly. All cases were followed routinely by our outpatient department for at least one year until the patient was lost to follow-up due to death, emigration to another district , or re-transplantation, whichever occurred first. Once serum bilirubin increased up to 2-fold of normal level, the patient was immediately admitted to hospital for further treatment.

### Statistics

Firstly, univariate analysis of risk factors which might be associated with BC was performed. Categorical variables were compared using the Chi-squared test. Mann-Whitney u-test was used to rank data and non-normal distribution continuous variables. According to univariate analysis and previous literature, all variables might be associated with BC were subjected to stepwise logistic regression analysis with 0.1 level for entry into the model . Odds ratios and 95% confidence intervals were calculated to filter out independent risks for BC.

Using cryoprecipitate transfusions as an exposure factor, the patients with intraoperative blood product transfusions were divided into two groups. A retrospective cohort study was carried out, and baseline fractures were compared between the two groups. Intraoperative blood loss was treated as the stratified factor of the two groups given it maybe a confounding factor., MH Chi-squared test was performed when analysis combined RR. Multivariate stepwise COX regression was also performed with 0.1 level for entry into the model, to enhance the risk evidence of BC. The BC-free survival curves were calculated according to the Kaplan–Meier method and compared using the log-rank test. The time between BC occurrence and obtaining of liver biopsies from BC patients were compared to detect the possible mechanism of BC occurrence.

Continuous data are presented as mean±standard deviation. All tests were two-sided. Statistical analysis was performed using the SPSS/PC Advanced Statistics Package, Version 19.0 (SPSS, Chicago, IL).Statistical tests were assumed to have reached significance at the conventional level of 0.05.

## Results

### Characters of BC patients and case-control analysis

In 356 patients, a total of 40 patients had developed the BC in the first year after LT, the overall incidence of BC was 11.2% (40/356). 356 patients were divided into two groups depending on whether they had developed BC or not. Pre-, intra- and postoperative factors, blood product transfusion are summarized in **TABLE 1** **.** The mean requirement of cryoprecipitate for the BC group was 13.5±12.2, while the non-BC group was 5.4±9.0 U (*P*<0.001). The need for RBC transfusion was significantly higher in BC group (10.2±8.9) than in non-BC group (8.1±10.6, *P* = 0.013). Univariate analysis also indicated that MELD (*P* = 0.017) and cold ischemia time (*P*<0.001), were statistically significant factors between the two groups. Furthermore, according to univariate analysis and previous literature, all variables might be associated with BC were subjected to stepwise logistic regression analysis to evaluate independent risk factors associated with BC. Multivariate logistic regression analysis demonstrated that cold ischemia time >8 h (OR = 6.30, 95% *CI* [2.97–13.3]), intraoperative cryoprecipitate transfusion (OR = 4.23, 95% *CI* [1.95–9.17]), and Child-Pugh (OR = 1.79, 95% *CI* [1.09–2.94]) were independent risk factors predicting BC after LT (**TABLE 2**).

**Table 1:** Patient characteristics and demographics by study groups.

Variables	Total	Non-BC	BC	P
	N = 356	N = 316 (88.8%)	N = 40 (11.2%)	
**Age(year)**	48±10	48±9	46±10	0.171
**Gender**				
Male	304 (85.4%)	269 (85.1%)	35 (87.5%)	0.689
Female	52 (14.6%)	47 (14.9%)	5 (12.5%)	
**Diagnosis**				
FHF*	45(12.6%)	40(12.7%)	5 (12.5%)	0.577
Cirrhosis	282(79.2%)	250 (79.1%)	32 (80.0%)	
Carcinoma	24 (6.7%)	22 (7.0%)	2 (5.0%)	
Others	5(1.4%)	4(1.3%)	1(2.5%)	
**Child-Pugh**				0.073
Grade A	117 (32.9%)	113(35.8%)	4 (10.0%)	
Grade B	142 (39.9%)	121 (35.4%)	21 (52.5%)	
Grade C	97 (27.2%)	82 (26.9%)	15 (37.5%)	
**ABO blood group**				
Compatible	306 (86.0%)	272 (86.1%)	34 (85.0%)	0.854
Incompatible	50 (14.0%)	44 (13.9%)	6 (15.0%)	
**MELD**				0.017
MELD≤10	53 (14.9%)	50(15.8%)	3 (7.5%)	
11≤MELD≤18	190 (53.4%)	175 (55.4%)	15 (37.5%)	
18<MELD≤24	20 (5.6%)	13 (4.1%)	7 (17.5%)	
MELD≥25	93 (26.1%)	78 (24.7%)	15 (37.5%)	
**Surgical factors**				
WIT* (min)	3.4±0.8	3.4±0.8	3.3±0.8	0.497
CIT* (min)	449±111	440±108	516±107	<0.001
Anhepatic phase (min)	58±10	58±10	58±7	0.578
Operation time (min)	392±95	389±90	411±130	0.851
Blood loss(ml)	3371±3419	3288±3451	4023±3121	0.025
Intravenous infusion(ml)	5890±2852	5893±2881	5869±2646	0.915
**Blood products transfusion**				
RBC(U)	8.3±10.4	8.1±10.6	10.2±8.9	0.013
FFP*(U)	2.0±4.7	1.9±4.4	2.8±6.5	0.86
PLT(U)	0.66±0.96	0.66±0.95	0.65±1.08	0.735
Cryo* (U)	6.3±9.7	5.4±9.0	13.5±12.2	<0.001
Whole blood(U)	0.40±2.07	0.38±2.10	0.55±1.92	0.172
Cell saver(ml)	573±1396	550±1391	754±1439	0.091
**Postoperative factors**				
**Immunesuppressor**				
FK506+MMF	305(85.7%)	270(85.4%)	35(87.5%)	0.595
CysA+MMF	43(12.1%)	38(12.0%)	5(12.5%)	
Others	8(2.2%)	8(2.5%)	0(0.0%)	
**Steroid**	195(54.8%)	172(48.3)	23(6.5%)	0.713
**Acute rejection**	7(2.0%)	6(1.7%)	1(0.3%)	0.569
**Chronic rejection**	9(2.5%)	6(1.7%)	3(0.8%)	0.068

* FHF = fulminant hepatic failure; FFP = fresh frozen plasma; WIT = warm ischemia time; CIT = cold ischemia time; Cryo = cryoprecipitate.

**Table 2:** Independent risk factors associated with BC (case-control analysis).

Variables	OR*	95% C.I.		P
		Lower	Upper	
Child-Pugh	1.79	1.09	2.94	0.022
CIT(>8 h)	6.30	2.97	13.3	<0.001
Cryo transfusion	4.23	1.95	9.17	<0.001

* OR were derived from multivariate stepwise logistic regression analysis. These factors were adjusted in the multivariate regression analysis: age, diagnosis, child-pugh, MELD, CIT, blood loss, RBC, Cryo transfusion, Cell saver transfusion, chronic rejection.

### Retrospective cohort analysis

We analyzed the incidence of BC by a retrospective cohort study. Stratified analysis was performed depending on whether a patient had blood loss of ≤2500 ml or >2500 ml (**TABLE 3**). Of the 221 patients with intraoperative blood loss of less than 2500 ml, the 60 patients that received intraoperative cryoprecipitate transfusions showed a higher BC incidence than the 161 patients who had no cryoprecipitate transfused (15.0% vs. 4.97%, RR = 3.02; 95% *CI* [1.22–7.46]; *P* = 0.013). Similarly, of the 135 patients with intraoperative blood loss more than 2500 ml, the 86 patients with cryoprecipitate transfused had significantly higher BC occurrence compared to the patients who did not receive cryoprecipitate (23.3% vs. 6.12%, RR = 3.80; 95% *CI* [1.19–12.1]; *P* = 0.011). When treated blood loss as the stratified factor, the combined RR of BC (Cryo vs no-Cryo) is 3.38(95% *CI* [1.62–7.05]; *P*<0.001). We then stratified patients according to the blood loss amount and compared the characteristics of the patients between intraoperative cryoprecipitate transfusion (cryo) or no-cryo groups (**TABLE 4**). For patients with less than 2500 ml blood loss, gender, diagnosis, MELD, RBC, FFP and Child-Pugh were found to be significantly different between cryo and no-cryo groups. However, for patients with more than 2500 ml blood loss, none of these characters were found to be significantly different.

**Table 3:** Incidence of BC in Cryo group and No-Cryo group.

	BC	RR*	95% C.I.		P
		Cryo vs No-cryo	Lower	Upper	
**Blood loss≤2500**		3.02	1.22	7.46	0.013
Cryo	9/60(15.00%)				
No-Cryo	8/161(4.97%)				
**Blood loss>2500**		3.80	1.19	12.1	0.011
Cryo	20/86(23.3%)				
No-cryo	3/49(6.12%)				
**Combined**		3.38	1.62	7.05	<0.001

* Univariate analysis was performed, the combined RR is computed when blood loss as the stratified factor.

**Table 4:** Baseline in No-cryo group versus cryo group.

	Blood loss≤2500 ml				Blood loss>2500 ml			
Variables	Total	Cryo	No-cryo	P	Total	Cryo	No-cryo	P
	N = 221	N = 60	N = 161		N = 135	N = 86	N = 49	
**Age(year)**	47.0±9.8	47.4±10.0	46.9±9.7	0.904	49.0±9.2	49.2±8.9	48.5±9.7	0.773
**Gender**				0.029				0.943
Male	197(89.1%)	49(81.7%)	148(91.9%)		107(79.3%)	68(79.1%)	39(79.6%)	
Female	24(10.9%)	11(18.7%)	13(8.1%)		28(20.7%)	18(30.9%)	10(20.4%)	
**Diagnosis**				0.035				0.322
FHF	13(5.9%)	5(8.3%)	8(5.0%)		32(23.7%)	22(16.3%)	10(20.4%)	
Cirrhosis	186(84.2%)	54(90.0%)	132(82%)		96(71.1%)	61(45.2%)	35(71.4%)	
Carcinoma	20(9.0%)	0(0%)	20(12.4%)		4(3.0%)	1(1.2%)	3(6.2%)	
Others	2(0.9%)	1(1.7%)	1(0.6%)		3(2.2%)	2(2.3%)	1(2.0%)	
**Child-Pugh**				0.001				0.105
**Grade A**	95(43.0%)	16(26.7%)	79(49.1%)		22(16.3%)	17(19.8%)	5(10.2%)	
**Grade B**	83(37.6%)	26(43.3%)	57(35.4%)		59(43.7%)	40(46.5%)	19(38.8%)	
**Grade C**	43(19.5%)	18(30.0%)	25(15.5%)		54(40.0%)	29(33.7%)	25(51.0%)	
**ABO blood group**				0.198				0.759
Compatible	192(86.9%)	55(91.7%)	137(85.1%)		114(84.4%)	72(83.7%)	42(85.7%)	
Incompatible	29(13.1%)	5(8.3%)	24 (14.9%)		21(15.6%)	14(16.3%)	7(14.3%)	0.810
**MELD**				0.041				0.079
MELD≤10	46(20.8%)	8(13.3%)	38(23.6%)		7(5.2%)	7(8.14%)	0(0%)	
11≤MELD≤18	122(55.2%)	31(51.7%)	91(56.5%)		68(50.4%)	45(52.3%)	23(46.9%)	
18<MELD≤24	12(5.4%)	3(5.0%)	9(5.6%)		8(5.9%)	6(7.0%)	2(4.1%)	
MELD≥25	41(18.6%)	18(30.0%)	23(14.3%)		52(38.5%)	28(32.6%)	24(49.0%)	
**Surgical factors**								
WIT (min)	3.4±0.8	3.3±0.8	3.4±0.8	0.510	3.4±0.8	3.3±0.8	3.4±0.8	0.654
CIT (min)	442±113	445±96	441±119	0.525	458±107	452±108	471±106	0.250
Anhepatic phase (min)	57.2±10.9	57.7±10.1	57.0±11.2	0.316	59.2±8.6	60.6±8.8	58.4±8.4	0.112
Operation time (min)	360±66	363±72	359±64	0.803	445±111	446±122	443±89	0.547
Intravenous infusion(ml)	4927±1359	4872±1402	4940±1347	0.915	7476±3800	7147±3738	8053±3878	0.079
**Blood products**								
RBC(U)	3.3±3.2	4.8±3.3	2.8±3.1	<0.01	16.5±12.7	17.2±12.1	15.2±13.7	0.132
FFP(U)	0.8±2.1	1.3±2.9	0.6±1.6	0.045	4.0±6.7	4.5±7.4	3.1±5.3	0.299
PLT(U)	0.4±0.8	0.4±0.8	0.4±0.8	0.859	1.2±1.1	1.1±1.1	1.1±1.1	0.910
Whole blood(U)	0.3±1.3	0.50±2.0	0.2±1.0	0.445	0.6±2.9	0.2±1.7	1.2±4.3	0.107
Cell saver(ml)	607+1350	594±1348	628±1358	0.659	1296±2038	1346±2184	1207±1772	0.749
**Postoperative factors**								
**Immunesuppressor**				0.060				0.093
FK506+MMF	188(85.1%)	55(91.7%)	133(82.6%)		117(86.7%)	75(87.2%)	42(85.7%)	
CysA+MMF	29(13.1%)	3(5.0%)	26(16.2%)		14(10.4%)	7(8.1%)	7(14.3%)	
Others	4(1.8)	2(3.33%)	2(1.2%)		4(3.0%)	4(4.7%)	0(0%)	
**Steroid**	118(53.4%)	35(58.3%)	83(51.6%)	0.808	77(57.0%)	45(52.3%)	32(65.3%)	0.143
**Acute rejection**	4(1.8%)	2(3.3%)	2(1.2%)	0.297	3(2.2%)	3(3.5%)	0(0.0%)	0.553
**Chronic rejection**	2(0.9%)	2(3.3%)	0(0%)	0.073	7(5.2%)	3(3.5%)	4(8.2%)	0.255

Further multivariate COX regression were performed to fix the difference of characteristics. This analysis showed that there was independent higher risk of BC when cold ischemia time >8 h (RR = 4.24, 95% *CI* [2.28–7.92], *P*<0.01), intraoperative cryoprecipitate transfusion (RR = 3.462, 95% *CI* [1.721–6.966], *P*<0.01), and high-level Child-Pugh (RR = 1.71, 95% CI [1.11–2.63], *P* = 0.014) after LT (**TABLE 5**). Therefore, the independent risk factors derived from cohort analysis were in accordance with case-control analysis.

**Table 5:** Independent risk factors associated with BC (cohort analysis).

Variables	RR*	95% C.I.		P
		Lower	Upper	
Cryo vs No-cryo	3.46	1.72	6.97	<0.01
CIT(>8 h) vs CIT(≤8 h)	4.24	2.28	7.92	<0.01
Child-Pugh increased one grade	1.71	1.11	2.63	0.014
Chronic rejection vs No chronic rejection	3.23	0.99	10.6	0.052

* RR were derived from multivariate stepwise COX regression.

### Pathological feature

All 37 liver biopsy specimens submitted from the BC patients were evaluated in this study. The biopsies showed pathological findings that ranged from nearly normal to severe cholestasis (**TABLE 6**). Varying degrees of inflammatory cell infiltration was seen in both groups. In most of the no-cryoprecipitate patients, the structure of the hepatic lobule was integrated (7/8), hepatic cells showed vacuolar degeneration (4/8), and some degree of epithelial hyperplasia was seen (4/8) (**Figure 1 A,C**). In comparison, in a majority of biopsies from the cryoprecipitate transfusion group, the integrity of the lobular structure was lost (21/29), part of the intrahepatic bile duct disappeared (19/29), and varying degrees of cholestasis and micro-thrombosis were observed in various sized portal area vessels (18/29, 16/29 respectively) (**Figure 1 B,D**).

**Figure 1:** Liver biopsies from BC patients. Representative histopathology images of BC patients liver biopsies, A,C are from No-cryo group and B,D are from Cryo group. In the No-cryo group, the structure of hepatic lobule was integrated, normal hepatic plates were observed, hepatic cells occurred vacuolar degeneration, bile duct epithelium hyperplasia and a few inflammatory cells infiltration, cholestasis was seen (**A, C**). The integrity of the lobular structure was loss. Intrahepatic bile ducts proliferated significantly, part of the bile duct disappeared. Bile duct epithelial deformation, atrophy, shedding, ?the portal area shows infiltration of lymphocytes, the intrahepatic seen varying degrees of cholestasis, micro-thrombosis was observed in various sized portal area vessels (**B, D**).

**Table 6:** Histopathological Features of Liver Biopsies from 37 BC patients.

Features	No-cryo	Cryo
	N = 8	N = 29
**Knodell HAI score** *		
Minimal (1–3)	3 ( 37.5%)	10 (34.5%)
Mild (4–6)	2 (25.0%)	12 (41.4%)
Moderate (7–9)	1 (12.5%)	4 (13.8%)
Marked (10–12)	0 ( 0%)	2 (6.9%)
**Hepatic lobule structure**		
Integrated	7 ( 87.5%)	8 (27.6%)
Disappeared	1 ( 12.5%)	21 (72.4%)
**Hepatic cells Vacuolar degeneration**	4 ( 50%)	9 (31.0%)
**Bile duct**		
Epithelial hyperplasia	4 ( 50%)	6 (20.7%)
Bile duct disappeared	1 ( 12.5%)	19 (65.5%)
**Cholestasis**	1 ( 12.5%)	18 (62.1%)
**Micro-thrombosis**	0 ( 0%)	12 (41.4%)

* Total of Knodell Histology Activity Index scores for periportal injury, parenchymal injury, and portal inflammation.

### Analysis of one year BC-free survival

The BC-free survival curve for post-transplant patients is shown in **Figure 2**. It shows that the BC-free survival rate for patients received intraoperative cryoprecipitate transfusions was significantly lower than the group that received no cryoprecipitate (*P*<0.001). According to previous literature, BC can be classified as early or late based on whether they occur ≤90 days or >90 days after LT [11]. The analysis of 40 patients who developed BC showed that, in the group receiving cryoprecipitate transfusion, BC occurred 111±84 days after LT and 18 out of 29 patients developed late BC. In the no-cryoprecipitate transfusion group, the mean time to BC occurrence was 72±59 days (*P* = 0.226) and 5 in 11 patients developed late BC (*P* = 0.477) (**TABLE 7**). Neither of these parameters was significantly different, indicating that the cryoprecipitate transfusion didn't alter the basic pathological properties of BC.

**Figure 2:** One year BC-free survival curve for live-transplant patients. One year BC-free survival curve for live-transplant patients according to the Kaplan–Meier method. BC-free survival probability of Patients received intraoperative cryoprecipitate transfusions(red line) was statistically significant lower when compared to the group that received no cryoprecipitate (blue line)(*P*<0.001).

**Table 7:** Analysis of BC occurrence.

Variables	Total	No-cryo	Cryo	P
	N = 40	N = 11	N = 29	
**Occurrence time (days)**	101±79	72±58.5	111±84	0.226
**Periods** *				0.477
Early BC	17 (42.5%)	6( 54.5%)	11 (37.9%)	
Late BC	23 (57.5%)	5 (45.5%)	18 (62.1%)	

* Periods classified based on the time of BC occurrence (Early BC occurred≤90 days after the operation, Late BC occurred >90 days after the operation).

## Discussion

Although BC is a major cause of graft loss and re-transplantation in patients who survive the early post-operative period after LT, the pathogenesis of BC is uncertain. In the last few years, multiple studies have found an association between intraoperative blood products transfusion and subsequently poor outcomes for patients who underwent LT [12]–[15]. Cryoprecipitate, which can control bleeding in LT through supplementation of fibrinogen and some pro-coagulant factors, was widely used in many centers. However, our study has shown that intraoperative cryoprecipitate transfusion was associated with the incidence of BC after LT. This result implies that cryoprecipitate transfusion during LTx should be performed only after careful consideration. Although our study did not provide a causal relationship between cryoprecipitate transfusion and BC, our analysis (case-control and cohort analysis) all indicated that cryoprecipitate transfusion is a significant risk factor of BC. Furthermore, it should be noted that while several baseline characters between cryo and no-cryo groups were significantly different in patients lost less than 2500 ml blood, none of these baseline characters were significantly different in patients lost more than 2500 ml blood (TABLE 4). This further supported the notion that cryoprecipitate transfusion is a significant risk factor, especially for patients lost more than 2500 ml blood.

The preparation of cryoprecipitate was first described by Judith Graham Pool in 1964 [16]. Cryoprecipitate is comprised of plasma coagulation proteins, in particular factor VIII, fibrinogen, von Willebrand factor, and Platelet microparticles (PMPs) [17]. The PMPs concentration of the cryoprecipitate has been shown to be 265-fold greater than that of the original plasma sample [18]. Isolated PMPs have been reported to activate both the extrinsic and intrinsic coagulation cascades [19], and provide a surface for thrombin formation [20]. Generally, PMPs have 50- to 100-fold higher specific procoagulant activity than activated platelets [21]. Therefore, cryoprecipitate might have a strong potential ability of promoting thrombosis. In the current study, micro-thrombus formation was observed more frequently in various sized portal area vessels in the massive cryoprecipitate transfusion group. This indicated that cryoprecipitate transfusion in LT might mediate the formation of micro-thrombosis.Large number of micro-thrombosis result in biliary microcirculation disturbance, leading to the occurrence of BC.

Small amounts of immunogenic components, such as immunoglobulin (IgG, IgM), are also present in cryoprecipitate [22]. In addition, previous research reported that PMPs are also capable of stimulating antigen-specific IgG production and activating adaptive immune cells [23]. When cryoprecipitate was transfused in patients underwent LT, the effects of these immune components were not take into account. In the current study, liver biopsy specimens from BC patients showed that bile ducts disappeared more frequently in cryoprecipitate transfusion group. As this pathological finding was one of the typical manifestations in organ rejection, it is strongly suggested that immunogenic components existed in cryoprecipitate, played an important role in the development of BC.

Despite the complex composition of cryoprecipitate, in end-stage liver disease patients, the criteria for when and how to use cryoprecipitate in LT has not been established. The British Committee for Standards in Hematology, Blood Transfusion Task Force and College of American Pathologists(CAP) have published guidelines for the use of cryoprecipitate, and is considered appropriate to use when the fibrinogen level was less than 1.0 g/L [24]–[26]. However, compared to healthy individuals, the coagulation system in patients with end-stage liver disease has its own characteristics. Both prohemostatic drivers and antihemostatic drivers in these patients are relatively reduced, and the entire coagulation system is a low-equilibrium state [27]. Moreover, end-stage liver disease patients are characterized by increased levels of factor VIII and von Willebrand factor combined with decreased levels of most other procoagulant factors [28]. Therefore, inappropriate cryoprecipitate transfusion to replenish fibrinogen can tip this fragile balance toward thrombosis simultaneously, due to high concentration of factor VIII, and von Willebrand factor contained in cryoprecipitate [17]. Once the thrombus formation affected the blood supply of biliary tract, the incidence of BC increased significantly. Furthermore , the fibrinogen content in a unit of cryoprecipitate varied widely, ranging from 120 to 796 mg [22], this was another important cause increased the degree of difficulty to use cryoprecipitate correctly.

In the current study, cold ischemia time more than 8 h is also associated with the incidence of BC. Many previous study have showed the same conclusion [29]–[31]. Although this finding was not new, it strengthened a concept that minimizing cold ischemic time is essential to reduce the risk of BC. Another study stressed that high MELD score might also contribute to the risk of BC [32], but our multivariate logistic regression analysis indicated that Child-Pugh classification, not MELD score, could be associated with the risk for BC. Previous study had also stressed certain MELD components (bilirubin level and international normalized ratio) to be risk factors for BC [33]. Therefore, recipient preoperative liver function trends might have effects on BC following LT, but further confirmation is required.

Previous literature has mentioned many other risk factors that may affect the incidence of BC, such as cytomegalovirus infection [34], Rh-incompatible [35], hepatitis C virus infection [36], and hepatic artery thrombosis [37]. However, these factors were relatively minimized in this research, and the relationship between the above factors and BC could not be further determined. In addition, some studies have also proposed that T tube drainages increased the incidence of BC [38], [39]. In our center, a randomized and controlled multicenter trial in 2001 reached the conclusion that T-tube drainages increased the incidence of BC [40], after which the T-tube drainages in LT had been abandoned. According to previous literature [11], we analyzed the time of BC occurrence, but there was no significant difference between cryoprecipitate transfusion group and no-cryoprecipitate transfusion group.

The limitation of the study was its retrospective nature. We did not evaluate factors that were not found for BC in the analysis. Surgical factors also contributed to the BC, but the role of these factors is becoming less significant due to the improvement of surgical techniques and perioperative care. Furthermore, we have no effective methods to carry out the assessment of the impact of surgical factors. So in this study, we excluded cases with biliary anastomosis strictures and vascular anastomotic stenosis, which were mainly caused by surgical techniques, and then the overall BC rate reduced to 11.2%.

The findings of our study suggested that cryoprecipitate transfusion, which was not noticed in other multiple analysis programs, was associated with the incidence of BC after LT. The possible risks of cryoprecipitate transfusions could be due to the complex ingredients in the product, which may cause micro-thrombus formation and immune rejection injury of bile ducts. To evaluate the exact role of cryoprecipitate transfusion playing in patients with end-stage liver diseases undergone LT, more randomized, controlled multicenter trials and further research needs to be performed to develop a reasonable, standard application regarding the use of cryoprecipitate in LT. Before this research is conducted, it is necessary to be cautious while using cryoprecipitate transfusions during LT. If the use of cryoprecipitate was solely for fibrinogen supplement, it is better to adopt the protocol carried out in some European countries, where cryoprecipitate was substituted by virally inactivated fibrinogen concentrate with more standardized concentration and a safer profile (effectively reducing the risk of pathogen and immune-related complications) [41], [42].
